# Surgery and Postoperative Care of Patients Undergoing Percutaneous Nephrolithotomy under the Guidance of B-Ultrasound Based on Smart Internet of Things

**DOI:** 10.1155/2022/8902195

**Published:** 2022-10-03

**Authors:** Hongyan Niu, Wei Li

**Affiliations:** ^1^Operating Room, The First Affiliated Hospital of Shandong First Medical University & Shandong Provincial Qianfoshan Hospital, Jinan, 250014 Shandong, China; ^2^Urology Surgery Department, The First Affiliated Hospital of Shandong First Medical University & Shandong Provincial Qianfoshan Hospital, Jinan, 250014 Shandong, China

## Abstract

At present, percutaneous nephrolithotomy has become an option for hospitals increasingly to treat calculus. However, due to the certain risk of percutaneous nephrolithotomy, it may lead to postoperative complications. Analyzing the preoperative factors of septic shock after percutaneous nephrolithotomy can provide guidance for reducing the incidence of septic shock after PCNL. This article establishes a logistic regression model based on preoperative factors, uses statistical methods, and uses the professional statistical software SPSS to create a database and analyze the data. The method of classification data analysis was used to determine various influencing factors including patient factors, stone factor, and preoperative factors and combined B-ultrasound guidance and percutaneous nephrolithotomy to reduce the risk of surgery. The experimental results found that the percutaneous nephroscope laser lithotripsy guided by the smart Internet of Things can effectively perform lithotripsy; in this paper, the preoperative data of different complications are obtained, and the risk of surgery is closely related to the operation time. The operation time exceeds 90 minutes and causes the risk of severe bleeding after PCNL. It is twice the operation time of less than 90 minutes and 5 times the operation time of less than 60 minutes.

## 1. Introduction

Clinically, upper urinary tract stones are part of urinary tract stones. The main treatment options include extracorporeal shock wave (ESWL), ureteroscopic lithotripsy (URL), and percutaneous nephrolithotomy (PCNL), and according to the characteristics and part, consider the appropriate treatment method. At present, PCNL has been widely used in the treatment of large and hard kidney stones, especially refractory kidney stones (staghorn stones, hard stones, stones with abnormal kidney anatomy, and stones for which other noninvasive treatments have failed). Although PCNL is considered a safe and effective minimally invasive stone removal procedure, complications still occur during work. Under normal circumstances, the bleeding can be stopped by conservative treatments such as immunosuppression, hemostatic drugs, and supplements. A small amount of bleeding can even be life-threatening, requiring renal artery accumulation or blood transfusion surgery. Therefore, the massive bleeding caused by PCNL should arouse the attention of urologists. Understanding the root cause of acute bleeding after PCNL has important clinical significance in preventing bleeding.

Before and after PCNL surgery, it is a common choice to determine the status of the patient's stones by B-ultrasound. To improve the operational efficiency, this article is aimed at combining the Internet of Things with B-mode ultrasound. The Internet of Things can establish the connection between things and things and things and communication networks through cognitive technology, network technology, communication technology, and embedded technology and capture, extract, measure, and distribute data through other data collection tools. There are many changes in this kind of data collection. As long as it is something that can be felt, its data can be collected and recognized by the server. The Internet of Things can also use cloud computing, information processing technology, data extraction, and other technologies for intelligent arithmetic and data information analysis. In traditional lithotripsy and lithotripsy operations, it is difficult to accurately determine the location of the calculi, and because the patient's case, body, and other factors are different, it is easy to cause problems during the operation. However, under the guidance of B-ultrasound based on the intelligent Internet of Things, the stone can be stably removed, and the patient's life is the main factor to ensure that it is carried out in a safe situation. The patient's situation can also be analyzed to obtain the best stone removal plan.

Regarding the treatment of stones, domestic and foreign experts have many studies. Santiago discussed the factors that affect the results during ureteroscopy (URS) and laser lithotripsy (LL) and discussed the specific clinical challenges of the efficacy of URS LL. URS LL has a high stone clearance rate in all locations of the urinary tract and all stone types and sizes. Comparing the data of LL and dust removal and basketry shows that the proportion of residual debris after dust removal is higher, but the utilization rate of the ureteral access sheath is lower, and the operation time may be shorter [1]. Mahmood compared the effectiveness and complications of holmium laser lithotripsy and pneumatic lithotripsy in the treatment of ureteral stones. Comparing 100 patients with ureteral calculi, the data show that holmium:YAG lithotripsy is safer and more effective than pneumatic lithotripsy in terms of immediate stone-free rate. The article believes that YAG is an excellent treatment for ureteral stones [2]. Yang evaluated the clinical efficacy and safety of holmium laser technology and extracorporeal shock wave lithotripsy (ESWL) combined with ureteroscopic lithotripsy (URSL) in the treatment of ureteral stones through a systematic review. Forest plots, sensitivity analysis, and bias analysis were carried out on the included articles. Summarized estimates of hazard ratio and standard mean deviation (SMD) and 95% CI are used as measures of effect size [3]. Different experts have different opinions on the prognosis of stones. Hochberger believes that more than 90% of common bile duct stones can be removed by endoscopic retrograde approach, endoscopic incision, and balloon catheter removal or mechanical lithotripsy. Laser lithotripsy represents a promising new endoscopic method. At present, only short-pulse laser systems with high peak power but low possibility of thermal damage to tissues are used for lithotripsy. Compared with extracorporeal shock wave therapy, laser lithotripsy can be performed in any endoscope unit within the pretreatment range of the endoscope [4]. Hendriks believes that due to mechanical obstruction caused by gallstones entering the gastrointestinal tract, stones larger than 2 cm may enter the digestive tract, which mainly occurs in the terminal ileum. Endoscope removal is the preferred technique. The advantage of using laser lithotripsy is that the energy can be accurately positioned on the stone while minimizing tissue damage [5]. Yang summarized the experience of percutaneous holmium laser lithotripsy in the treatment of bladder stones with lower urinary tract obstruction or pelvic arthropathy and explored its efficacy and safety. It is concluded that percutaneous holmium laser lithotripsy is an improved minimally invasive surgical technique for the treatment of bladder stones. It has the advantages of clear surgical field, high stone retrieval efficiency, small trauma, low pressure of bladder perfusion, auxiliary injury, and low incidence of infection [6]. Sun compares the different effects of two-shift and single-shift flexible ureteroscope holmium laser lithotripsy for the treatment of kidney stones larger than 1.5 cm on surgical results and operator comfort. Flexible ureteroscope holmium laser lithotripsy is used to treat kidney stones larger than 1.5 cm. The two-shift operation can improve the speed of lithotripsy and stone removal rate, significantly reduce the fatigue of the operator, and improve the comfort of the operator [7]. These studies provide some references for this article, but due to insufficient data in related studies and missing samples, the results of the experiment are difficult to reproduce and unconvincing.

The innovation of this paper is to take stones from patients through B-ultrasound under the intelligent Internet of Things, and the postoperative patients with septic shock as the research object. According to the collected data, the appropriate influencing factors are screened out and established, logistic regression model is used for multivariate analysis, and finally the analysis results are acquired, to provide guidance for reducing the incidence of septic shock after PCNL and provide reference for subsequent research.

## 2. Laser Lithotripsy and Nursing Methods

### 2.1. Smart Internet of Things

The Internet of Things can be explained as with the help of information technologies such as laser monitors, global positioning systems, infrared sensors, and radio frequency identification (RFID), according to various procedures to determine the integration of objects connected to the IT network on the data platform to complete the data and information interactive network to understand the understanding of established sites and operations [8]. Through the Internet of Things, smart medical care can be realized. IoT refers to the use of technologies such as information sensing, RFID, GPS, infrared, and laser scanning. Objects or programs can collect all required information, such as optical, thermal, electrical, mechanical, chemical, biological, and location, and use various networks to obtain information, with the ability to intelligently recognize, identify, and manage projects and processes. The Internet of Things is a network based on the Internet and traditional telecommunication networks, which links all common physical objects that can be located independently.

Smart Medical integrates all account resources of medical companies to form a source pool. The user makes an appointment through the Internet and visits the hospital at the appointment time, which not only saves the patient's time but also avoids the overcrowding of the family and the difficulty of curing. Through the hospital APP, WeChat, employee number, and other channels, users can perform tasks such as paying for medical cards, paying for medical expenses, and viewing test reports, which simplifies the patient's medical treatment process, and users do not need to queue back and forth for different hospitals and charging windows [9]. The Internet of Things is shown in Figure 1.

For the smart Internet of Things, the first thing to estimate is whether the economic benefits that can be obtained after the system is implemented and the test is successfully deployed and whether the cost of the system development process is reasonable [10, 11]. If the R&D cost is too high relative to the economic benefits of the subsequent system and the system is not sufficiently forward-looking to be a cornerstone for future project launches, then the starting point of the project's system R&D will have a big problem. The startup is debatable. If the technical difficulty required for the realization of the system is too large, difficult to maintain, or even difficult to develop in the future, it will lead to a long R&D cycle, which will affect the revenue that the system can bring and the formation of a black hole in R&D costs; the consequences will be unimaginable [12]. The overall scheme architecture of the system is shown in Figure 2.

The artificial intelligence medical expert diagnosis is to use the realized medical diagnosis expert system to simulate the diagnosis of the user's symptoms by the human expert so that the patient and the user can know the symptoms of the user, and it is also convenient for the expert to communicate more effectively during the face-to-face consultation, which is conducive to the expert's decision [13]. The medical expert system is a computer program that collects, organizes, and analyzes a large number of cases by computer, concentrates the diagnosis results of medical experts, and can diagnose a certain disease. By reasoning about rules, cases, mathematics, and neural networks, simulations are performed through fault recovery techniques and image scanning methods. For some minor diseases diagnosed without going to medical institutions for treatment, users can also take simple treatment measures, which also reduces the waste of valuable medical resources, reduces the difficulty of medical institutions, and makes the limited resources better serve the society [14].

If there is a need for face-to-face consultation after diagnosis, the user can make an online appointment according to the reference symptoms given by the system. And you can check your appointment at any time and check the report after the inspection.

### 2.2. B-Ultrasound Image Denoise

The position noise can be described by a multiplier noise model, because the influence of the compression transformer on the B-mode image must be considered. For the B-ultrasound image model, the fidelity constraint item is improved, and the uniqueness of the model solution in the space. The gradient method used in this paper is slower to ensure that the model is a convex model [15].

The upper and lower limits of the solution are estimated as frame constraints, combined with the Split Bregman algorithm, a corresponding fast algorithm is proposed, and the convergence result of the algorithm is given. After adopting the Split Bregman algorithm, the quality of the obtained image will be significantly improved, and the information degree of the image will be guaranteed, and the pixel distribution will be uniform and have better contrast. Finally, simulation experiments verify the feasibility and effectiveness of the algorithm [16]. A new fidelity term model is proposed to process medical images in B-mode:

(1) $$\begin{array}{c} E_{1}\left(u\right)=\int_{\Omega }\frac{{\left(u-f\right)}^{2}}{u}. \end{array}$$

Combining the ROF model and the fidelity term, the following model is proposed:

(2) $$\begin{array}{c} \underset{u}{\min}\left\{\int_{\Omega }\left|Du\right|+\lambda \int_{\Omega }\frac{{\left(f-u\right)}^{2}}{u}\right\}. \end{array}$$

Among them, *λ* ≥ 0 is the weight parameter. And the theoretical analysis of the existence and uniqueness of the model solution in the BV space is given, but the gradient descent method used in this article is relatively slow and has hard requirements *λ* ≥ 0. Therefore,

(3) $$\begin{array}{c} E\left(u\right)=\underset{u}{\min}\left\{\int_{\Omega }\left.\left|Du\right|+\lambda \int_{\Omega }\frac{{\left(f-u\right)}^{2}}{u}\right)\right\}. \end{array}$$

The Split Bregman algorithm transforms the complex problem solving into solving several easy subproblems. For example, the following constraint problem:

(4) $$\begin{array}{c} \min\int_{\Omega }\left|\overset{⟶}{d}\right|dx+\lambda \int_{\Omega }F\left(z,f\right)dx. \end{array}$$

The following solution to the problem is called in each iteration:

(5) $$\begin{array}{c} \min\int_{\Omega }\left|\overset{⟶}{d}\right|dx+\lambda \int_{\Omega }F\left(z,f\right)dx+\frac{y_{1}}{2}\left\|\overset{⟶}{d}-Du-\overset{⟶}{b}1\right\|+\frac{y_{2}}{2}. \end{array}$$

The two newly added items are secondary penalty items, ${\overset{⟶}{b}}_{1}$ and the sum *b*_2_ is a variable. Fix *z* and *u* to minimize *d*, then fix *d* and *u* to minimize *z*, and so on. Three subproblems were formed.

First, for the subproblem of *d*, fix *z* and *u* as follows:

(6) $$\begin{array}{c} \min\int_{\Omega }\left|\overset{⟶}{d}\right|dx+\frac{y_{1}}{2}\left\|\overset{⟶}{d}-Du-{\overset{⟶}{b}}_{1}\right\|. \end{array}$$

It can draw

(7) $$\begin{array}{c} {\overset{⟶}{d}}^{k+1}\left(x\right)=\frac{{Du}^{k}\left(x\right)+b_{1}^{k}\left(x\right)}{\left|{Du}^{k}\left(x\right)+b_{1}^{k}\left(x\right)\right|}\max\left\{{Du}^{k}\left(x\right)+b_{1}^{k}\left(x\right)\left|-1y_{1},0\right.\right\}. \end{array}$$

Secondly, for the problem of *z*, fix *d* and *u* as follows:

(8) $$\begin{array}{c} \underset{z}{\min}\lambda \int_{\Omega }F\left(z,f\right)dx+\frac{y_{2}}{2}. \end{array}$$

Then, *z* satisfies

(9) $$\begin{array}{c} \lambda \partial_{z}F\left(z,f\right)+y_{2}\left(z-u-b_{2}\right)=0. \end{array}$$

Equation (9) represents the condition that *z* needs to satisfy to minimize *d*. *z* is a fixed factor.

For Gaussian white noise

(10) $$\begin{array}{c} F\left(z,f\right)=\frac{1}{2}{\left(z-f\right)}^{2}. \end{array}$$

Equation (10) represents the Gaussian white noise in the case of *z* minimum. So

(11) $$\begin{array}{c} z\left(x\right)=\frac{u\left(x\right)+b_{2}\left(x\right)+\left(\lambda /y_{2}\right)f\left(x\right)}{1+\left(\lambda /y_{2}\right)}. \end{array}$$

Finally, for the problem of *u*, fix *d* and *z* as follows:

(12) $$\begin{array}{c} \underset{u}{\min}\frac{y_{1}}{2}{\left\|\overset{⟶}{d}-Du-b_{1}\right\|}_{2}^{2}+\frac{y_{2}}{2}{\left\|z-u-b_{2}\right\|}_{2}^{2}. \end{array}$$

Then, *u* satisfies

(13) $$\begin{array}{c} \frac{y_{2}}{y_{1}}u-\Delta u=\frac{y_{2}}{y_{1}}\left(z-b_{2}\right)-\mathrm{div}\left(\overset{⟶}{d}-{\overset{⟶}{b}}_{1}\right). \end{array}$$

Use fast Fourier transform to find *u*:

(14) $$\begin{array}{c} {\overset{\wedge }{u}}^{k+1}=\frac{\left(y_{2}/y_{1}\right)\left(z^{k+1}-b_{2}^{k}\right)-\left(\mathrm{div}\left(d^{k+1}\right)b_{1}^{k}\right)}{\left(y_{2}/y_{1}\right)-\hat{\Delta }}. \end{array}$$

The training set contains *M* training samples, and the sigmoid function is selected as the output function; then,

(15) $$\begin{array}{c} Q_{pi}=f\left(u_{pi}\right)=\frac{1}{1+\exp\left(-u_{pi}\right)}. \end{array}$$

Among them, *Q*_*pj*_ is the output of neuron *j*, and *W*_*ji*_ is the weight of neuron *j* to neuron *i*.

Suppose the network error function is *E*; then,

(16) $$\begin{array}{c} E_{p}=\frac{1}{2}\overset{1}{\underset{i=0}{\sum }}{\left(d_{pi}-O_{pi}\right)}^{2}. \end{array}$$

Among them, M is the number of samples, *E*_*p*_ was the error of the *p*-th sample, and the expected output of neuron *i*.

Using the gradient descent method, to enable the weight to change along the negative gradient direction of the error function, set the weight change as then

(17) $$\begin{array}{c} \Delta W_{ij}={\eta \delta }_{pi}O_{pi},\;\eta \geq 0. \end{array}$$

Among them, *η* is the learning factor and *δ*_*pi*_ is the error term. Because the function has *f*′(*x*) = *f*(*x*)(1 − *f*(*x*)), the result is

(18) $$\begin{array}{c} \Delta w_{jk}=-\eta \left(d_{i}-y_{i}\right)y_{i}\left(1-y_{i}\right){\text{net}}_{j}. \end{array}$$

A certain mean compensation is required for the predicted value, and the EWMA (Exponential Weighted Moving Average) algorithm is used for compensation.

(19) $$\begin{array}{c} {\bar{X}}_{t}\left(h\right)=\lambda X_{t}\left(h-1\right)+\left(1-\lambda \right)\frac{1}{t_{N}}. \end{array}$$

Therefore, the expression can be obtained as

(20) $$\begin{array}{c} X_{t}\left(h\right)=-\overset{\infty }{\underset{k=1}{\sum }}g\left(k\right)X_{t}\left(h-k\right)+\overset{p}{\underset{i=1}{\sum }}\varphi_{i}. \end{array}$$

Generally, ordinary images have a relatively large dynamic range, and the gray values of pixels are evenly distributed in the entire gray range. Therefore, intuitively, the entire image will have a relatively high contrast, and the details can be seen very clearly [17, 18]. The image demanipulation process is shown in Figure 3.

The histogram balance method is based on the analysis of the above principles. Specifically, the histogram equation is to operate the image gray level histogram to improve the image quality. The main method is to increase the dynamic range of the total grayscale pixel value so that the narrow grayscale range in the original image can be extended to a relatively uniform distribution of the entire grayscale, so the overall contrast of the image will also be improved, respectively [19].

### 2.3. Preoperative Preparation and Postoperative Prognosis

Whether the patient has serious bleeding diseases before the operation, such as hemophilia and idiopathic thrombocytopenic purpura syndrome, the bleeding risk of such diseases is very high, and it will be difficult to control the bleeding after operation. It should be listed as an absolute contraindication of the operation and must be treated in relevant departments. In addition, some patients with serious cardiopulmonary diseases cannot tolerate surgery, and patients with acute infection and renal tuberculosis should not be operated immediately [20]. Many systemic system diseases that affect coagulation function may also be related factors that cause bleeding, such as diabetes, hypertension, and syndrome X.

The common causes of bleeding after PCNL are the violent and frequent activities of getting out of bed early and the premature removal of the nephrostomy tube. In addition, when the patient has constipation or coughing activity after the operation, the intra-abdominal pressure will suddenly increase, which may cause the newly formed blood scab to fall off and cause rebleeding [21]. Another factor is that the small arteries and venules in the kidney are more or less damaged during the operation, which may lead to the formation of pseudoaneurysms, arteriovenous fistulas, and eventually bleeding. If the necessary measures are not taken, it will cause severe bleeding.

PCNL needs to establish percutaneous renal channels, which will undoubtedly bring substantial damage to the kidney and then have varying degrees of bleeding. In our daily clinical work, we should take preventive measures for patients with such bleeding. In case of massive bleeding, we should timely carry out a reasonable and effective clinical intervention [22]. The blood vessels can be coagulated with electrocautery or the blood vessels can be ligated, or the bleeding can be stopped by compression.

Once it is determined that the patient is bleeding during PCNL surgery, the severity of the bleeding should be judged, and then, appropriate treatment interventions should be taken: when the amount of bleeding is small, hemostatic drugs can be used, and when the bleeding affects the function, the work may be temporarily stopped and shut down [23]. If the bleeding site is found under direct observation of bipolar electrocoagulation or laser, the bleeding can also be stopped. Once the bleeding stops, the operation can be continued. If the above method is invalid and there is still a lot of bleeding during the operation, the operation should be stopped and the second operation should be selected. Tighten to increase the internal pressure of the collection system to force the bleeding to stop.

In summary, there are many related factors that cause bleeding after PCNL, including the patient's own factors and the clinical operation of the operator. It is of great clinical significance to explore and understand the key risk factors of severe bleeding after PCNL, and it can provide certain help to prevent and reduce severe bleeding after surgery. Because patients with stones are not as good as death every day, they need to endure a lot of suffering. In addition, there are methods to stop the bleeding during the operation, and the risk of bleeding can be reduced by controlling the operation time, which leads the patient to want to get rid of this pain and want to have the operation. At the same time, once we find a patient with severe postoperative bleeding, we should calm down and take reasonable and appropriate clinical interventions in a timely manner so that the bleeding can be effectively controlled.

This study included patients who were diagnosed with nephrolithiasis or ureteral pulmonary nodules in the Department of Urology at the City First Hospital from January 20, 2019 to December 2019. Patients who have no absolute surgical contraindications and are willing to receive PCNL treatment are as follows: preoperative white blood cells' total number is >12 × 10^9^/L or <4 × 10^9^/L; the patient's preoperative basic heart rate is >90 beats/min, and the basic body temperature is >38°C or <36°C. Long-term oral inhibitors are required. Before the operation, B-ultrasound, intravenous urography, and urinary tract computed tomography+three-dimensional reconstruction were performed to confirm the diagnosis and assess the degree of hydronephrosis and the size of the stones. The main brackets used during the operation are shown in Figure 4.

## 3. Lithotripsy Experiment and Results

### 3.1. Patient Information

In this paper, the patients after the diagnosis were tested in batches, and the patients were graded according to the physiological data information of the patients before surgery. To ensure the accuracy of the experiment, the experimental data were selected from 100 people at different levels. The hospital classifies the patient's information. Quantitative is to quantify the amount of drugs used before surgery and the situation of surgery. Qualitative is to qualitatively characterize the patient's condition and classify the nature of different diseases. Separate statistics are helpful for distinguishing different consequences of different situations and for subsequent judgments. The classified information mainly includes the patient's age, condition, history, and drug use time. The main information is shown in Table 1. The effects of fixed factors are mainly gender, whether there are other diseases, inflammation in the body, type, etc. Calculate according to the historical statistics of independent variables and dependent variables, and establish regression analysis equations on this basis, namely, regression analysis prediction model. Through the investigation of the patients in the questionnaire, the information in Table 2 was obtained according to the patient's condition. The results are shown in Table 2.

After the operation, the number of people who had intermittent sleep due to physical reasons was 8, accounting for 0.9% of the total patients. The hormone levels and drug levels in the patients were detected, but no specific cause was found. See Table 3 for details.

According to the calculation of the patient's urine data, the time of the patient's infection can be determined, see Table 4.

Logistic regression equation was used to set gender, age, history of diabetes, affected side, urine culture, urinary system infection, stone size, stone type, hydronephrosis, etc. This is due to septic shock. Urine culture and urinary tract infection remained the main risk factors after excluding mixed factors. *X*1: positive urine culture, see Figure 5; *X*2: surgery for urinary tract infection.

By obtaining the situation of model calculation, the prevalue of the model is calculated, and then, the corresponding data information is obtained by mathematical calculation method according to the dynamics of each group of data. The result is shown in Figure 6.

By judging the value of the reasons in the model for 10 different qualitative and quantitative situations, the probability of possible concurrency is judged according to these data situations and the graph under normal conditions. The higher the curve similarity, the higher the probability of concurrency.

### 3.2. Percutaneous Nephroscope Laser Lithotripsy

The patient first takes the bladder lithotomy position and disinfects it regularly, and then changes to the prone position to prepare for the operation. All patients undergoing PCNL surgery were guided by ultrasound, starting from the posterior axillary line to the affected scapular line. Under the guide wire, it will increase the peritoneal dilator. In the meantime, it should pay attention to the depth of expansion. Finally, the functional case extends to the renal pelvis, forming percutaneous renal lithotripsy and removal channels, as shown in Figure 7.

We have made statistics on the calculation factors of patients. Among the stone factors, multiple stones accounted for about 81.2% of the total number of patients, with 49 cases of severe bleeding after surgery. Patients with calculus diameters > 2 cm accounted for 56.0% of the total number of patients, and 33 cases had severe postoperative bleeding. Stones accounted for about 9.1% of the total number of patients, and 5 cases suffered severe bleeding after surgery. There were 325 cases of stones in the renal pelvis and calyces, accounting for 50.0% of the total number, and 39 cases of severe bleeding after surgery. There were 50 cases of kidney stones before operation, accounting for 50.0% of the total, and 39 cases of severe bleeding after operation. Through the analysis, it was found that the occurrence of severe postoperative bleeding in multiple kidney stones was related to the severity of the stones, as shown in Figure 8.

Statistically significant indicators of general condition (history of hypertension, diabetes history, preoperative coagulation function, renal insufficiency, urinary tract infection, and hydronephrosis) and upper urinary tract calculi were statistically significant indicators (renal calculus location) and operator factors (intraoperative channel number, single channel size, staging procedure, and operation time). Multivariate logistic regression was used for analysis. The results are shown in Figure 9.

It can be seen that the risk of severe bleeding after PCNL is 2.2 times higher than that of the microchannel during operation. The risk of severe bleeding after PCNL is 2.0 times higher than that of less than 90 min and 5.0 times higher than that of less than 60 min. The risk of severe bleeding after PCNL caused by preoperative urinary infection is 18.7 times higher than that without preoperative urinary infection, preoperative creatinine value > 115 *μ*mol/L, that is, the risk of severe bleeding after PCNL caused by renal insufficiency is 3.2 times higher than that without obvious abnormality of renal function.

If patients with conservative treatment have poor hemostasis or hemorrhage occurs, renal angiography should be performed in time, and SRAE treatment should be given. In this study, patients suffered from abdominal pain and other symptoms after surgery and found that there was bleeding and bleeding from the drainage tube of the renal fistula. If there is persistent gross hematuria in an emergency, the patient's family members were actively communicated, and after obtaining consent, SRAE was performed, and finally, the bleeding was controlled. Among patients undergoing renal artery angiography and embolization, hemorrhage was found in a branch vessel at the upper pole of the patient's renal artery during the operation, and hemorrhage in a branch vessel at the middle pole of the renal artery was found in the patient. The rest of the patients were all under renal artery bleeding from a branch of the pole. The preoperative and postoperative conditions of the patient that underwent SRAE are shown in Figure 10.

## 4. Discussion

At present, PCNL is generally used for the treatment of complex kidney stones and upper ureteral stones. At the same time, with the development of endourology, PCNL, especially in the treatment of large kidney stones (≥2 cm) and staghorn stones, has gradually become an indispensable surgical choice, which plays an important role and plays an increasingly important role. However, PCNL is not an absolutely safe operation, and there are still complications such as infection, bleeding, injury, and urinary leakage. Bleeding after PCNL is one of the common complications. In general, when most patients have postoperative bleeding, they can be stopped after conservative treatment, such as braking hemostatic drugs and blood transfusion. A few patients with a large amount of bleeding must undergo selective renal arteriography embolization. In severe cases, nephrectomy is required, and very few will lead to death.

To reduce the complications of PCNL in the treatment process, we combined B-ultrasound for treatment. PCNL ultrasound-guided B and standard PCNL channel laser lithotripsy lasers are both safe and effective, and each has advantages in clinical efficacy. Both MPCNL and standard PCNL channels have the advantages of less postoperative damage and fewer complications. The running time of the standard PCNL channel is shorter than that of MPCNL. The standard PCNL channel is suitable for larger kidney stones. For multiple stones, MPCNL should be considered first. Therefore, we will have to decide which surgical method to choose according to the specific situation of each patient, such as the size and distribution of the stones and the technical ability of the surgeon, and even combine the two surgical methods to achieve the best result.

In the experimental analysis of this study, it was found that there was a history of hypertension, a history of diabetes, abnormal preoperative freezing activity, preoperative creatinine value > 115 *μ*mol/L, which is the average value of renal failure, urinary tract infection, severe stone, and renal pelvic stones. However, at the same time, considering that the various observers will influence each other, if some indicators or factors are analyzed separately, there will be some shortcomings and limitations, and the overall components need to be fully considered. In addition, the analysis results should be effectively combined with the actual situation of clinical work, use professional knowledge to conduct reasonable analysis and discussion, eliminate lies, maintain the truth, and obtain risk factors with greater clinical guidance. Therefore, this study uses logistic multiple regression analysis to effectively correct and control the statistically significant indicators of factor analysis. The final result is that urinary tract infection, renal failure, large intraoperative puncture tube, and operation time exceeding 90 minutes are the main risk factors for severe bleeding after PCNL.

For patients with urinary tract infection, antibiotics should be used reasonably before operation to control urinary tract infection. For patients with high fever and other symptoms, nephrostomy can be performed before operation. After the body temperature drops to normal and the urine routine returns to negative, the stones can be treated by operation. For patients with viscous yellow purulent mass in the renal collecting system during operation, the operation should be terminated immediately, the nephrostomy tube should be given for drainage, and high-dose broad-spectrum antibiotics should be used. If necessary, bacterial culture should be done. Antibiotics should be applied according to the culture results. When the infection returns to negative, percutaneous nephrolithotripsy should be performed. The drainage of the fistula tube must be smooth after operation. In addition, for such patients, when using a nephrostomy tube, a certain dose of furosemide can also be injected intravenously to make the intrarenal pressure lower than the glomerular filtration pressure, which can maximize the extravasation of perfusion fluid, reduce the chance of reflux, and finally reduce the probability of bleeding and sepsis.

It is controversial whether patients with basic diseases such as hypertension and diabetes should undergo PCNL surgery routinely. The conclusions of whether hypertension and diabetes can contribute to bleeding after PCNL are not completely consistent. Therefore, in clinical work, to further increase the safety of the operation and the patient's trust in the doctor, it is found that patients with basic diseases such as hypertension and diabetes should use antihypertensive drugs and hypoglycemic drugs before PCNL surgery. Control the blood pressure and blood sugar level within the normal allowable range, and monitor the changes in blood pressure and blood sugar in the time after the operation. If operation patients with a large fluctuation range are found, they should be dealt with in time.

## 5. Conclusions

With the popularization of PCNL technology and the development of equipment, the operation is widely carried out in inpatients. The factors leading to severe bleeding after PCNL include many aspects, especially the general situation of patients, stone factors, and the clinical function of operators. The results of this study showed that history of hypertension, history of diabetes, preoperative coagulation dysfunction, preoperative creatinine value > 115 *μ*mol/L, namely, renal failure, urinary tract infection, moderate and severe hydronephrosis, multiple renal calculi, pelvic cavity hydronephrosis, multiple root canal, larger puncture tube, progressive operation, and operation time were statistically significant for severe bleeding after PCNL. Of course, this study also has some shortcomings. Because this study is a retrospective study, some defects and omissions will inevitably appear in the process of statistical data. Some indicators, such as antibiotic use history, infection history before treatment, data and information during hospitalization, and preoperative medication or placement of ureteral stents in other hospitals, may lead to deviations in statistical information. Therefore, there may be some errors in the final conclusion. In future research, it is necessary to strengthen the universality of samples and reduce experimental variables. The best experimental effect has been achieved.

## Figures and Tables

**Figure 1:** IoT.

**Figure 2:** System framework diagram.

**Figure 3:** Image denoising process.

**Figure 4:** Props used for percutaneous nephrolithotomy. (a) Uteroscope (used for microchannel Lithotripsy) (b) Percutaneous renal puncture kit.

**Figure 5:** Multivariate regression analysis of postoperative infection.

**Figure 6:** Goodness of fit test.

**Figure 7:** Percutaneous nephroscope laser lithotripsy guided by ultrasound.

**Figure 8:** Bleeding after calculus surgery.

**Figure 9:** Statistically significant indicators.

**Figure 10:** Comparison of patients before and after bleeding.

**Table 1:** General information of patients.

Variable	Minimum	Max	$\bar{x}\pm s$
Age	17	82	47 ± 12
Creatinine before operation (*μ*mmol/L)	17	1180	94 ± 79
Stone size (mm)	4	65.7	18.7 ± 7.9
Number of surgical channels	1	3	1.51 ± 0.3
Operation time (min)	14	149	62.1 ± 21.6
Antibiotic application days before surgery	1	16	3.5 ± 2.3

**Table 2:** Qualitative patient data.

Variable	Classification and assignment	Number of cases
Gender	1: female	357
	2: male	524
Generation	1: ≤60	217
	2: >60	509
History of preoperative diabetes	0: no	170
	1: yes	813
Affected side	1: left	428
	2: right	437
Positive urine culture	0: negative	736
	1: positive	143

**Table 3:** Preoperative data of different complications.

Variable	Complication		Statistic value	*P*
	Normal group	Complication group		
Age	48.75 ± 12.21	42.64 ± 17.31	0.862	0.263
Creatinine before operation (*μ*mmol/L)	94.37 ± 81.09	67.76 ± 19.89	0.464	0.127
Stone size (mm)	19.81 ± 8.79	21.46 ± 10.75	0.903	0.548
Number of surgical channels	1.42 ± 0.39	1.87 ± 0.24	0.353	0.897
Operation time (min)	59.01 ± 25.64	71.51 ± 24.4	0.944	0.132
Antibiotic application days before surgery	3.48 ± 2.32	5.14 ± 4.06	0.829	0.431

**Table 4:** Comparison of preoperative qualitative data of different complications.

Variable		Complication		Chi-square group	*P*
		Normal group	Complication group		
Gender	1: male	54	3	0.828	0.259
	2: female	39	4		
Generation	1: ≤60	45	2	2.761	0.214
	2: >60	48	5		
History of preoperative diabetes	0: no	64	6	0.066	0.784
	1: yes	29	1		
Affected side	1: left	45	3	0.33	0.981
	2: right	48	4		

## Data Availability

No datasets were analyzed during the current study.
